# Antibody immune responses and causal relationships in four immune skin diseases: Evidence from Mendelian randomization and Bayesian Weighting (Antibody Responses in Skin Diseases: MR & Bayesian)

**DOI:** 10.1111/srt.13875

**Published:** 2024-08-09

**Authors:** Xiaojian Li, Shiyu Chen, Yunbo Wu, Guirong Qiu, Shiping Cheng, Hongrong Lan, Zhangren Yan, Dongbei Huang

**Affiliations:** ^1^ Clinical Medical College Jiangxi University of Chinese Medicine Nanchang China; ^2^ Dermatology Department Affiliated Hospital of Jiangxi University of Chinese Medicine Nanchang China

**Keywords:** atopic dermatitis, *Helicobacter pylori*, immune response, Mendelian randomization, psoriasis, rosacea, vitiligo

## Abstract

**Background:**

Recent studies increasingly suggest that microbial infections and the immune responses they elicit play significant roles in the pathogenesis of chronic inflammatory skin diseases. This study uses Mendelian randomization (MR) and Bayesian weighted Mendelian randomization (BWMR) to explore the causal relationships between immune antibody responses and four common skin diseases: psoriasis, atopic dermatitis (AD), rosacea, and vitiligo.

**Methods:**

We utilized summary statistics from genome‐wide association studies (GWAS) for antibody responses to 13 infectious pathogens and four skin diseases. Single nucleotide polymorphisms (SNPs) were selected as instrumental variables (IVs) to assess causal relationships using multiple MR methods, including inverse variance weighted (IVW), MR Egger, and weighted median. BWMR was also employed to confirm findings and address potential pleiotropy.

**Results:**

The IVW analysis identified significant associations between specific antibody responses and the skin diseases studied. Key findings include protective associations of anti‐Epstein–Barr virus (EBV) IgG seropositivity and *Helicobacter pylori* UREA antibody levels with psoriasis and AD. anti‐chlamydia trachomatis IgG seropositivity, anti‐polyomavirus 2 IgG seropositivity, and varicella zoster virus glycoprotein E and I antibody levels were negatively associated with rosacea, while EBV Elevated levels of the early antigen (EA‐D) antibody levels and HHV‐6 IE1B antibody levels were positively associated with rosacea. *H. pylori* Catalase antibody levels were protectively associated with vitiligo, whereas anti‐herpes simplex virus 2 (HSV‐2) IgG seropositivity was positively associated with vitiligo. The BWMR analysis confirmed these associations.

**Conclusion:**

This study underscores the significant role of *H. pylori* and other pathogens in these skin diseases, suggesting both protective and exacerbating effects depending on the specific condition. Understanding these pathogen‐immune interactions can lead to the development of more effective, personalized treatments and preventative strategies, ultimately improving patient outcomes and quality of life.

## 1 INTRODUCTION

Skin diseases such as psoriasis, atopic dermatitis (AD), rosacea, and vitiligo are prevalent chronic inflammatory conditions globally. These ailments not only impair patients' quality of life but also precipitate substantial psychological stress and social challenges. Individuals with psoriasis frequently endure severe itching and pain, whereas those afflicted with AD are susceptible to infections due to excessively dry and fissured skin. Rosacea patients often suffer from diminished self‐esteem as a result of facial erythema and papules, while those with vitiligo may encounter social stigmatization and profound psychological distress due to depigmentation.^1^, ^2^, ^3^, ^4^ Although current research has made some progress in uncovering the causes and mechanisms of these diseases, their complex etiology and multifactorial nature still make their pathological mechanisms difficult to fully elucidate. The interplay of environmental factors, genetic predispositions, immune system abnormalities, and microbial infections presents significant challenges in the study and treatment of these conditions.^5^, ^6^

Recent evidence increasingly suggests that microbial infections and the immune responses they elicit play significant roles in the pathogenesis of these skin diseases. Studies have found that certain pathogens can not only directly infect skin cells but also influence disease progression through complex immune reactions.^7^, ^8^ For instance, infections with pathogens such as Epstein–Barr virus (EBV), human herpesvirus 6 (HHV‐6), *Helicobacter pylori*, polyomavirus, and herpes simplex virus type 2 (HSV‐2) have been reported to be associated with various immune‐related diseases. These pathogens can induce the host to produce specific antibodies, thereby affecting the balance of the immune system, and in some cases, triggering or alleviating skin diseases.^9^, ^10^ For example, EBV infection may modulate T‐cell function, impacting the development of psoriasis and AD; HHV‐6 might exacerbate rosacea symptoms through reactivation; and the antibody response induced by *H. pylori* infection could influence the progression of vitiligo through antioxidant pathways.^11^, ^12^ However, the specific relationships between antibody responses and skin diseases require further investigation.

This study aims to explore the relationships between 46 immune antibodies and four skin diseases—psoriasis, AD, rosacea, and vitiligo—using Mendelian randomization (MR) and Bayesian weighted analysis. MR is a method that uses genetic variation as IVs to assess causal relationships, effectively reducing the influence of confounding factors and reverse causation.^13^ Bayesian weighting, on the other hand, integrates data from different sources to provide more robust analytical results.^14^ By combining these advanced analytical methods, we hope to uncover causal relationships between immune antibody responses and skin diseases, thereby providing new insights and scientific evidence for the diagnosis, prevention, and personalized treatment of these diseases, and offering valuable references for clinical practice.

## 2 MATERIALS AND METHODS

### 2.1 Study design

In MR analysis, single nucleotide polymorphisms (SNPs) serve as IVs. These IVs need to meet three essential assumptions depicted in Figure 1: (1) a strong correlation between the SNP and the exposure; (2) no correlation between the SNP and any confounders that might affect the exposure‐outcome relationship; and (3) the SNP affects the outcome exclusively through the exposure.^15^

**FIGURE 1:** Plot of key assumptions for MR analysis. MR, Mendelian randomization.

### 2.2 Data sources

The GWAS conducted by Guillaume Butler‐Laporte^16^ provides summary statistics for the genome‐wide association of antibody responses to 13 infectious pathogens. This study evaluated the genetic basis of 46 phenotypes related to antibody‐mediated immune responses using the UK Biobank cohort (*n* = 8735 individuals). It identified multiple loci associated with these immune traits, including genome‐wide significant loci within the major histocompatibility complex (MHC) on chromosome 6 and 60 additional loci outside the MHC. Notable associations included those with EBV‐related non‐communicable diseases (such as loci at RASA3, MED12L, and IRF4) and polyomaviruses (with the FUT2 gene). The study also highlighted the significance of various HLA alleles, including DRB109:01, DQB102:01, DQA101:02, and DQA103:01 in EBV serology, and DRB1*15:01 in polyomavirus serology.

Summary statistics for four skin diseases were obtained from the FinnGen GWAS (https://r8.finngen.fi/). The numbers of cases and controls for each phenotype are as follows: psoriasis (6995 cases, 299 128 controls), AD (8281 cases, 278 635 controls), rosacea (1877 cases, 297 544 controls), vitiligo (191 cases, 291 889 controls), as detailed in the Table S1,S2.

### 2.3 Instrumental variable selection

SNPs robustly associated with the exposures were selected using a genome‐wide significance threshold of < 5.0×10^−8^. To eliminate linkage disequilibrium, an *r* ^2^ threshold of 0.001 and a clump window size of 10 000 kb were applied.^17^ The strength of the IVs was assessed using the *F*‐statistic, calculated as *F* = *β* ^2^/SE^2^, where *β* is the effect size of the allele and SE is the standard error.^18^ An *F*‐statistic greater than 10 indicates the absence of weak IV bias,^19^ as detailed in Table S3.

### 2.4 Statistical analysis

Using the selected IVs, two‐sample MR analyses were performed on the five skin diseases utilizing the TwoSampleMR and MRPRESSO packages in R (version 4.4.0). MR analysis was conducted using five methods: inverse‐variance weighted (IVW) as the primary method, supplemented by MR Egger, weighted median, simple mode, and weighted mode. The IVW method, which uses a meta‐analysis approach to combine the causal effect estimates from various SNPs, served as the basis for our analysis.^20^ MR Egger accounts for nonzero mean pleiotropy but has reduced statistical power.^21^ Weighted median provides robust estimates if at least 50% of the weight comes from valid IVs.^22^ A simple mode is a model‐based approach offering robustness to pleiotropy,^23^ while weighted mode is sensitive to heterogeneity.^24^

To further address “weak instrument and weak level pleiotropy,” Bayesian weighted Mendelian randomization (BWMR) was employed. The BWMR model considers the uncertainty due to polygenicity and addresses violations of IV assumptions due to pleiotropy using Bayesian‐weighted outlier detection.^14^

### 2.5 MR results

Our study found that anti‐EBV IgG seropositivity, EBV VCA p18 antibody levels, EBV ZEBRA antibody levels, Human herpes virus 6 IE1B antibody levels, *H. pylori* UREA antibody levels, and anti‐Merkel cell polyomavirus IgG seropositivity are significantly associated with psoriasis (*p* < 0.05), as details shown in Figure 2.

**FIGURE 2:** MR results of antibody immune responses and psoriasis. MR, Mendelian randomization.

Anti‐EBV IgG seropositivity, EBV virus VCA p18 antibody levels, EBV ZEBRA antibody levels, human herpes virus 6 IE1B antibody levels, *H. pylori* UREA antibody levels, and anti‐Merkel cell polyomavirus IgG seropositivity are significantly associated with AD (*p* < 0.05), as details shown in Figure 3.

**FIGURE 3:** MR results of antibody immune responses and AD. AD, atopic dermatitis; MR, Mendelian randomization.

Anti‐chlamydia trachomatis IgG seropositivity, EBV EA‐D antibody levels, EBV ZEBRA antibody levels, human herpes virus 6 IE1B antibody levels, anti‐polyomavirus 2 IgG seropositivity, and varicella zoster virus glycoproteins E and I antibody levels are significantly associated with rosacea (*p* < 0.05), as details shown in Figure 4.

**FIGURE 4:** MR results of antibody immune responses and rosacea. MR, Mendelian randomization.

EBV ZEBRA antibody levels, *H. pylori* catalase antibody levels, *H. pylori* VacA antibody levels, anti‐herpes simplex virus 2 (HSV‐2) IgG seropositivity, and anti‐polyomavirus 2 IgG seropositivity are significantly associated with vitiligo (*p* < 0.05), as details shown in Figure 5.

**FIGURE 5:** MR results of antibody immune responses and rosacea. MR, Mendelian randomization.

The specific SNP profiles for these four groups, as well as pleiotropy and heterogeneity results, can be found in Table S4. No evidence of pleiotropy was observed (*p* > 0.05). The *F*‐statistics for all groups were greater than 10, indicating no weak instrument bias. Table S4 shows the MR analysis involving these antibody immune responses and the four skin diseases. Notably, the heterogeneity test suggested some heterogeneity within groups (*p* < 0.05), prompting us to conduct a Bayesian weighted analysis.

### 2.6 BWMR results

Considering the presence of horizontal pleiotropy in some of the analysis results, we further employed BWMR for these groups. The BWMR analysis revealed the following significant associations (Figures 6 and 7), as detailed in the Table S5:

1. Psoriasis: anti‐EBV IgG seropositivity and *H. pylori* UREA antibody levels.
2. AD: anti‐EBV IgG seropositivity and *H. pylori* UREA antibody levels.
3. Rosacea: anti‐chlamydia trachomatis IgG seropositivity, EBV EA‐D antibody levels, human herpes virus 6 IE1B antibody levels, anti‐polyomavirus 2 IgG seropositivity, and varicella zoster virus glycoproteins E and I antibody levels.
4. Vitiligo: *H. pylori* Catalase antibody levels and HSV‐2 IgG seropositivity.
5. After applying the Bayesian weighting, these associations remained significant (*p* < 0.05).

**FIGURE 6:** Bayesian weighted Mendelian randomization results.

**FIGURE 7:** Scatterplot.

## 3 DISCUSSION

Recent studies have increasingly demonstrated that microbial infections and the subsequent immune responses play a critical role in the pathogenesis of chronic inflammatory skin diseases.^25^, ^26^ In this study, MR was employed to comprehensively investigate the causal relationships between immune antibody responses and four common skin diseases: psoriasis, AD, rosacea, and vitiligo. This was followed by BWMR for further validation, thereby providing robust evidence to support future research endeavors.

First, our study found that anti‐EBV IgG seropositivity and *H. pylori* UREA antibody levels are significantly negatively associated with psoriasis (*p* < 0.05). This finding suggests that EBV infection and *H. pylori* infection may play protective roles in the pathogenesis of psoriasis. EBV is a common herpesvirus with a widespread global prevalence. After EBV infection, the host immune system generates IgG antibodies against the virus, which can persist in the body long‐term.^27^ Studies show that EBV infection can promote the differentiation and expansion of Tregs by upregulating the expression of certain cytokines such as IL‐10 and TGF‐β. These Tregs can inhibit the function of effector T cells and reduce the release of inflammatory mediators, thereby alleviating the symptoms of psoriasis to some extent.^28^

*H. pylori* is a bacterium that can infect the gastric mucosa, and elevated UREA antibody levels are negatively correlated with psoriasis.^29^ *H. pylori* infection typically triggers a chronic inflammatory response but can also suppress excessive immune reactions by inducing the production of regulatory T cells (Tregs).^30^ Specifically, after *H. pylori* infection, the host immune system may reduce psoriasis‐related inflammatory responses by modulating specific inflammatory pathways. This mechanism may include inhibiting the production of pro‐inflammatory cytokines or balancing the immune response by increasing the levels of anti‐inflammatory cytokines.^31^

It is interesting to note that anti‐EBV IgG seropositivity and *H. pylori* UREA antibody levels also have a significant negative correlation with AD. Similar to psoriasis, after EBV infection, the host immune system produces IgG antibodies, which may alleviate the symptoms of AD by modulating the immune response.^32^ For example, EBV‐specific IgG antibodies may be involved in regulating the function of T cells, including promoting the differentiation and function of Tregs, which can suppress excessive immune responses and the release of inflammatory mediators.^33^

*H. pylori* infection can induce the production of UREA antibodies, which may be associated with the alleviation of AD symptoms. *H. pylori* infection typically triggers chronic inflammation, but it can also suppress excessive immune reactions by inducing the production of Tregs. This immune regulation may reduce AD‐related inflammatory responses by inhibiting the production of pro‐inflammatory cytokines or by increasing the levels of anti‐inflammatory cytokines.^34^

For rosacea, MR studies have found significant associations with anti‐chlamydia trachomatis IgG seropositivity, EBV EA‐D antibody levels, Human herpes virus 6 IE1B antibody levels, anti‐polyomavirus 2 IgG seropositivity, and varicella zoster virus glycoproteins E and I antibody levels. Among these, EBV EA‐D antibody levels and Human herpes virus 6 IE1B antibody levels are positively correlated with rosacea, while anti‐chlamydia trachomatis IgG seropositivity, anti‐polyomavirus 2 IgG seropositivity, and varicella zoster virus glycoproteins E and I antibody levels are negatively correlated with rosacea.

EBV is a ubiquitous herpesvirus that can infect B lymphocytes and epithelial cells.^27^ Elevated levels of the early antigen (EA‐D) typically indicate an active infection by the virus. EBV may cause rosacea by inducing a chronic inflammatory response in the host's immune system.^35^, ^36^ Increased activity of EBV could lead to the immune system releasing more pro‐inflammatory cytokines, such as IL‐6 and TNF‐α, thereby exacerbating skin inflammation.

HHV‐6 is also a human herpesvirus that primarily infects T lymphocytes. Elevated levels of HHV‐6 IE1B antibodies suggest the reactivation of the virus. Studies indicate that HHV‐6 can trigger chronic inflammatory responses through various pathways, including the activation of inflammatory cytokines and chemokines, which may lead to the exacerbation of rosacea symptoms.^37^

Chlamydia trachomatis is a pathogen that causes sexually transmitted diseases, commonly resulting in reproductive system infections such as urethritis, cervicitis, and pelvic inflammatory disease.^38^ After infection, the human immune system responds to the pathogen by producing specific IgG antibodies against Chlamydia trachomatis. The presence of IgG antibodies typically indicates that the host has been previously infected with the pathogen and has developed a certain degree of immune memory.^39^ Studies have shown that chlamydial infection can induce the immune system to produce anti‐inflammatory cytokines, such as IL‐10 and TGF‐β. These anti‐inflammatory cytokines can suppress excessive inflammatory responses, protecting tissues from damage.^38^ For patients with rosacea, chronic inflammation is one of the main factors exacerbating the condition. The anti‐inflammatory cytokines induced by chlamydial infection may reduce skin inflammation, thereby lowering the risk of developing rosacea.

Polyomavirus 2, also known as JC virus, is a widespread virus that typically reactivates when the immune system is suppressed. A positive IgG antibody indicates past infection and suggests that the individual may have some level of immune memory. Interestingly, some studies suggest that after Polyomavirus 2 infection, the regulation of the host immune system might provide cross‐protection against other pathogen infections, which could potentially reduce the risk of rosacea.^40^

After infection with the varicella‐zoster virus (VZV), the immune system typically generates long‐term memory antibodies. The E and I glycoproteins of VZV are major antigenic components of the virus, and elevated levels of IgG antibodies may help reduce inflammatory responses in rosacea by modulating the immune system.^41^ This effect could be related to the immune system's cross‐reactivity to VZV antigens or the suppression of specific inflammatory pathways.^42^ In the context of rosacea, chronic inflammation is a key factor that exacerbates the condition. VZV‐specific antibodies, particularly IgG, may regulate the immune response to lessen the severity of inflammation associated with rosacea. This could be due to an enhanced ability of the immune system to recognize and respond to VZV antigens, leading to a more regulated inflammatory response.^42^ Additionally, the cross‐reactivity of memory T cells to other pathogens might play a role in reducing the risk of rosacea flare‐ups.

Finally, there is a significant association between *H. pylori* Catalase antibody levels and HSV‐2 IgG seropositivity with vitiligo. There is a significant negative correlation between *H. pylori* Catalase antibody levels and vitiligo, while there is a significant positive correlation between HSV‐2 IgG seropositivity and vitiligo.

Infection with *H. pylori* triggers an immune response in the host, leading to the production of antibodies targeting Catalase. This enzyme plays a crucial role in antioxidant defense by breaking down hydrogen peroxide, a reactive oxygen species, thus mitigating oxidative stress.^43^ Oxidative stress is notably higher in individuals suffering from vitiligo,^44^ a skin condition characterized by the loss of melanocytes, the cells responsible for producing skin pigment. The increased antibody levels against *H. pylori* Catalase may suggest an enhanced antioxidant mechanism in the host, which could help in reducing oxidative damage to melanocytes. This protective mechanism might contribute to the prevention or slowing down of vitiligo progression.^45^, ^46^

Regarding the positive correlation between HSV‐2 IgG Seropositivity and vitiligo, current research does not offer a definitive mechanism. However, we can speculate on some potential connections. An HSV‐2 infection typically triggers an immune response that produces specific IgG antibodies. This immune response may lead to inflammation and changes in immune regulation, which could affect the skin's melanocytes.^47^ For instance, the inflammatory response might release cytokines and chemokines that could damage or destroy melanocytes, thereby causing vitiligo. Additionally, an HSV‐2 infection might activate underlying autoimmune processes. In some cases, the immune response to a viral infection could cause the body to attack its own tissues, which might affect melanocytes and consequently lead to the development of vitiligo.^48^

### 3.1 Strengths and limitations

This study utilized advanced analytical methods such as MR and BWMR, which effectively reduce the influence of confounding factors and reverse causation, providing more reliable causal inferences. The research covers four common chronic inflammatory skin diseases: psoriasis, AD, rosacea, and vitiligo, offering comprehensive pathological mechanism explorations with high clinical application value. Additionally, the study delves into the relationships between different pathogen infections and immune responses, particularly highlighting the multifaceted role of *H. pylori* in various skin diseases, providing new perspectives for understanding the complex etiology of skin diseases. The data sources are extensive, utilizing large‐scale genomic data from the UK Biobank and FinnGen GWAS, which have broad representativeness and high statistical power, enhancing the reliability of the research results.

However, despite the ability of MR to reduce some confounding factors, the study is still based on observational data, which may have potential biases that have not been fully eliminated. Although the research explored multiple pathogens, the in‐depth study and mechanism exploration of certain specific pathogens might still be insufficient, requiring further experimental validation and clinical research support. Despite the wide‐ranging data sources, they are primarily based on genomic data from European populations, potentially limiting the applicability to other ethnic groups and regions, thus requiring cautious extrapolation of the results. Additionally, the study is based on single time‐point antibody levels and genotype data, lacking dynamic observation of changes in pathogen infections and immune responses on disease progression over time. Overall, this study has significant advantages in revealing the causal relationships between immune antibody responses and skin diseases, but it also has some limitations that need further validation and refinement in future research.

## 4 CONCLUSION

In conclusion, this comprehensive analysis provides novel insights into the causal relationships between immune antibody responses and four immune‐related skin diseases. By leveraging advanced analytical methods such as MR and BWMR, our findings offer a more robust understanding of the etiological roles of various pathogens in psoriasis, AD, rosacea, and vitiligo. Our study underscores the significant role of *H. pylori* in these skin diseases, suggesting that its infection might have both protective and exacerbating effects depending on the specific condition. Understanding these pathogen‐immune interactions can lead to the development of more effective, personalized treatments and preventative strategies, ultimately improving patient outcomes and quality of life.

Future research should focus on elucidating the specific immune pathways involved in these associations and exploring potential therapeutic interventions targeting these immune responses. The findings from this study provide a strong foundation for future investigations and highlight the importance of considering microbial infections in the context of chronic inflammatory skin diseases.

## CONFLICT OF INTEREST STATEMENT

The authors declare no commercial or financial ties that could be perceived as a conflict of interest.

## ETHICS STATEMENT

This study did not require ethical approval because all data were sourced from publicly available databases. Written consent from participants was not needed as this complies with national legislation and legal policies.

## Supporting information

Supporting Information

## Data Availability

Datasets analyzed in this study can be found in The biobankengine at https://biobankengine.stanford.edu/ and the FinnGen repository at https://r8.finngen.fi/.
